# Relationship between Neutrophil Gelatinase-Associated Lipocalin, Eosinophil Cationic Protein, Cytokines, and Atopic Sensitization in Patients with Allergic Diseases

**DOI:** 10.1155/2022/6564706

**Published:** 2022-06-06

**Authors:** Jong Weon Choi, Moon Hee Lee, Tatsuyoshi Fujii

**Affiliations:** ^1^Department of Laboratory Medicine, College of Medicine, Inha University, Incheon, Republic of Korea; ^2^Department of Internal Medicine, College of Medicine, Inha University, Incheon, Republic of Korea; ^3^Department of Internal Medicine, Tsukuba University Hospital Mito Clinical Education and Training Center, Mito Kyodo General Hospital, Ibaraki, Japan

## Abstract

The effect of neutrophil gelatinase-associated lipocalin (NGAL) on eosinophil activation, atopic sensitization, and systemic inflammation in allergic diseases has rarely been investigated. This study aimed to investigate the relationship between NGAL, eosinophil cationic protein (ECP), cytokines, and allergen-specific immunoglobulin E (sIgE) in allergic diseases. A total of 136 patients with allergies and 58 healthy individuals were evaluated. The concentrations of NGAL, ECP, tumor necrosis factor-*α* (TNF-*α*), interleukin-5 (IL-5), sIgE, total IgE (tIgE), and high-sensitivity C-reactive protein (hsCRP) were measured. The transforming growth factor-*β*1 (TGF-*β*1) level was measured as a profibrotic marker of bronchial asthma. Allergic patients had significantly higher NGAL, ECP, and hsCRP levels than healthy individuals. However, there was no significant difference in NGAL levels between patients with positive and negative ECP tests and those with high and low sIgE scores. Asthmatic patients with elevated NGAL exhibited a significantly higher TGF-*β*1 level than those without elevated NGAL. However, no significant difference was observed in the ECP, IL-5, and sIgE levels between the two groups. Among the patients with a positive ECP test, subjects with elevated hsCRP had two times higher NGAL levels than those without elevated hsCRP. NGAL was positively correlated with TNF-*α*, TGF-*β*1, and hsCRP, but not with ECP, IL-5, tIgE, and sIgE. An elevated NGAL level led to a 1.3-fold increase in the prevalence of high TGF-*β*1 (odds ratio: 1.31; 95% CI: 1.04–2.58; *P* < 0.001). In conclusion, NGAL elevation may be more closely linked to allergic inflammation and a possible fibrotic change in the airways than to the severity of eosinophil activation and atopic sensitization.

## 1. Introduction

Allergic diseases are a group of immune-mediated illnesses characterized by a hyper-responsiveness of the immune system to environmental antigens [1]. They are primarily caused by the interaction of an allergen with its specific immunoglobulin E (sIgE) on the surface of mast cells, which leads to the secretion of chemical mediators that induce the production of inflammatory cells [2]. According to the type of allergy and the target organ of contact with allergens, various clinical manifestations can occur in the airways, skin, or gastrointestinal tract, such as bronchial asthma, urticaria, eczema, vomiting, and diarrhea [3].

Eosinophil cationic protein (ECP) is a cytotoxic protein present in the protein matrix of eosinophils [4]. ECP is released from the secondary granules of activated eosinophils and is largely responsible for damaging the bronchial mucosa [5]. ECP is closely related to allergic diseases and contributes to airway inflammation observed in these diseases. During the progression of allergic diseases, ECP, released locally from the inflamed mucosa, infuses into the circulating blood, resulting in systemic inflammation [6].

Neutrophil gelatinase-associated lipocalin (NGAL), also called lipocalin-2, is a 25 kDa glycoprotein associated with neutrophilic inflammation. NGAL is known as an acute phase protein because its blood level is increased under various inflamed conditions [7]. NGAL was initially identified as a matrix protein of specific granules of human neutrophils but later found to be secreted by different cells, including renal tubular cells, immune cells, and respiratory epithelial cells [8]. As extracellular matrix proteins play an important role in the process of airway remodeling, NGAL has been regarded as a potential indicator of airway structural alteration in patients with pulmonary diseases [9]. However, there have been conflicting results on NGAL in patients with allergies. In some studies, NGAL was significantly elevated in patients with bronchial asthma and chronic obstructive pulmonary disease (COPD) [10, 11]. However, in another study, there was no significant difference in NGAL levels between asthmatic patients and healthy individuals [12].

Previous studies of NGAL have mainly focused on the clinical use of NGAL as an indicator of acute kidney injury [13] or as a predictor for the progression of chronic kidney disease [14]. There are few studies on NGAL production and its relationship with ECP, sIgE, cytokines, and inflammatory parameters in allergic diseases [10–12]. Therefore, this study investigated whether plasma NGAL is elevated in allergic diseases in proportion to the severity of eosinophil activation and atopic sensitization. This study also evaluated the association between NGAL and fibrotic changes in the airways by measuring the level of transforming growth factor-*β*1 (TGF-*β*1), which is a promising profibrotic biomarker of airway remodeling in bronchial asthma.

## 2. Materials and Methods

### 2.1. Subjects

This cross-sectional study was conducted in 136 patients (71 men and 65 women) who were diagnosed with allergic diseases. Age- and sex-matched healthy individuals (*n* = 58) without any evidence of allergy and inflammation were enrolled as the control group. The patients' age ranged from 20 to 72 years (mean age: 50.2 years). Subjects with confirmed allergy were chosen based on the following criteria: a clinical history of allergic reaction, elevated serum total IgE (tIgE) level, and positive sIgE tests for inhalant and/or food allergens according to the ImmunoCAP assay. The patients had the following diseases: bronchial asthma (*n* = 83), food allergy (*n* = 31), allergic rhinitis (*n* = 12), atopic dermatitis (*n* = 5), allergic conjunctivitis (*n* = 3), and anaphylaxis (*n* = 2). The mean duration of allergies was 1.4 years, and 75 (55.1%) patients had a history of allergic attack (Table 1). Several parameters, including NGAL, ECP, interleukin-5 (IL-5), tumor necrosis factor-*α* (TNF-*α*), TGF-*β*1, sIgE, tIgE, and high-sensitivity C-reactive protein (hsCRP) levels, were measured. The following subjects were excluded from the study to avoid the effects of their diseases on ECP and NGAL levels: (a) those with medication history, including corticosteroids or histamine antagonists; (b) those with acute infection with fever, chronic illness, and recent surgery; and (c) those with renal dysfunction, cardiovascular diseases, and sepsis. Subjects with missing values in medical records and fasting time <8 h were also excluded from the analysis. Information on the status of cigarette smoking was obtained. The study protocol was approved by the Institutional Review Board of Inha University Hospital (approval number: 2021-06-002). This study was performed following the guidelines of the Helsinki Declaration. Subjects were categorized into several groups according to the NGAL, ECP, ECP/eosinophil (ECP/Eo) ratio, and sIgE levels: elevated NGAL (*n* = 56) and nonelevated NGAL (*n* = 80); positive ECP test (*n* = 110) and negative ECP test (*n* = 26); elevated ECP/Eo ratio (*n* = 68) and nonelevated ECP/Eo ratio (*n* = 68); and high sIgE score (*n* = 86) and low sIgE score (*n* = 50). Patients with positive ECP test were further stratified into two groups based on the hsCRP level: elevated hsCRP (*n* = 69) and nonelevated hsCRP (*n* = 41).

### 2.2. Measurement of Laboratory Parameters

Blood samples were drawn from patients at the first visit to the hospital and collected in vacutainer tubes. All specimens were collected prior to treatment. Samples were centrifuged at 2500×*g* for 20 min and immediately analyzed for the following parameters: hsCRP, IgE, ECP, and NGAL. For the measurement of cytokines, samples were stored at -80°C until analysis. The concentration of NGAL was measured by fluorescence immunoassay using the Triage NGAL test kit (Alere Inc., San Diego, CA, USA). The cutoff value of plasma NGAL was set at 150 ng/mL [15]. Serum ECP was analyzed by chemiluminescent immunometric assay using an Immulite 2000 analyzer (Siemens Healthcare Diagnostics, Tarrytown, NY, USA). An elevated ECP level above 19 *μ*g/L was regarded as positive [16]. The ECP/Eo ratio was calculated with the following equation: ECP/Eo ratio = serum ECP level (*μ*g/L)/blood eosinophil count (/*μ*L). An elevated ECP/Eo ratio was defined as >0.24, which was a provisional cutoff limit based on the median level of the ECP/Eo ratio of the patient populations. The sIgE test for inhalant allergens (*Dermatophagoides farinae* and *Dermatophagoides pteronyssinus*) and food allergens (cow's milk and egg white) was performed using a fluoroenzyme immunoassay (ImmunoCAP 100, Phadia AB, Uppsala, Sweden). An sIgE level ≥0.35 kU/L, namely, ≥class I, was defined as allergic sensitization [17]. The sIgE score was obtained by the summation of the class, which was given to each patient according to the grade of allergic sensitization. High and low scores of sIgE were determined as >3 and ≤3, respectively, based on the median sIgE level of the allergic patients. The concentration of tIgE was measured using an immunoradiometric assay (Coat-A-Count Total IgE IRMA, Siemens Healthcare Diagnostics, Tarrytown, NY, USA). The concentrations of IL-5, TNF-*α*, and TGF-*β*1 were measured using enzyme-linked immunosorbent assay kits (R&D Systems, Minneapolis, MN, USA; BD Inc., San Diego, CA, USA; and RayBiotech, Norcross, GA, USA, respectively) according to the manufacturer's instructions. As a profibrotic marker of the airways, TGF-*β*1 was measured only in patients with bronchial asthma. The hsCRP level was measured using a particle-enhanced immunonephelometric assay with a chemical analyzer (Hitachi 7600; Hitachi, Tokyo, Japan). An elevation of hsCRP level was defined as >0.5 mg/dL, which was based on the cutoff value (95% confidence interval) for hsCRP levels in healthy individuals. Blood eosinophil counts were estimated using an automated analyzer (ADVIA 120; Siemens, Forchheim, Germany).

### 2.3. Statistical Analysis

Data were expressed as mean ± standard deviation (SD) or median (interquartile range: IQR). Categorical variables were presented as frequency and percentage. The normality of data was tested by the Kolmogorov-Smirnov test. Continuous variables with normal distribution were analyzed by Student *t* test. Nonnormally distributed data were analyzed by the Mann–Whitney *U* test. The chi-square test was used to analyze categorical variables. The relationship between NGAL, ECP, cytokines, and allergy-related parameters was assessed by multivariate linear regression analysis with adjustment for potential confounders, such as age, sex, body mass index (BMI), systolic blood pressure (SBP), and current smoking. The association between elevated NGAL and the prevalence of high TGF-*β*1 was evaluated by multivariate logistic regression analysis. Statistical analysis was performed with the SPSS software package (version 26; IBM SPSS Statistics, Armonk, NY, USA) and the MedCalc software package (version 20; MedCalc Software Ltd., Ostend, Belgium). Values of *P* < 0.05 were considered statistically significant.

## 3. Results

### 3.1. Characteristics of Subjects

ECP, tIgE, sIgE, and the ECP/Eo ratio were significantly higher in allergic patients than in healthy individuals. Of the 136 patients, 56 (41.2%) patients had elevated NGAL levels, and 91 (66.9%) patients had elevated hsCRP levels (Table 2). The NGAL level of the allergic patients was 137.5 ng/mL, significantly higher than that (69.5 ng/mL) of the control subjects (*P* < 0.001) (Figure 1).

### 3.2. NGAL in Allergic Patients with and without Systemic Inflammation

The NGAL level of allergic patients with systemic inflammation was significantly higher than that of allergic patients without systemic inflammation (152.3 ng/mL vs 86.7 ng/mL, *P* < 0.001). However, there was no significant difference in the NGAL levels between allergic patients without systemic inflammation and healthy individuals. Patients with systemic inflammation exhibited higher ECP/Eo ratios than those without systemic inflammation; however, no significant difference in ECP, tIgE, and sIgE levels was observed between the two groups (Table 3).

### 3.3. ECP and Cytokines in Patients with Elevated NGAL

Patients with elevated NGAL had significantly higher TNF-*α*, TGF-*β*1, and hsCRP levels than those without elevated NGAL (71.5 pg/mL, 3.52 ng/mL, and 2.13 mg/dL vs 30.8 pg/mL, 1.87 ng/mL, and 0.45 mg/dL, respectively, *P* < 0.001). However, there was no significant difference in ECP, IL-5, the ECP/Eo ratio, and sIgE levels between the groups (Table 4).

### 3.4. NGAL and Cytokines according to ECP and the ECP/Eo Ratio

Compared to patients with a negative ECP test, those with a positive ECP test had significantly higher IL-5, tIgE, and sIgE levels. Similarly, patients with elevated ECP/Eo ratios had higher levels of the corresponding parameters than those without elevated ECP/Eo ratios (*P* < 0.001). However, no significant differences in NGAL and TGF-*β*1 levels were observed between patients with positive and negative ECP tests or between patients with and without elevated ECP/Eo ratios (Table 5).

### 3.5. ECP and NGAL according to sIgE and hsCRP Levels

ECP and the ECP/Eo ratio were significantly higher in patients with a high sIgE score than in those with a low sIgE score. However, no significant difference was observed in NGAL and proinflammatory cytokine levels between the two groups. The plasma NGAL level was two-fold higher in patients with a positive ECP test and elevated hsCRP than in those with a positive ECP test and nonelevated hsCRP (181.5 ng/mL vs 90.2 ng/mL, *P* < 0.001) (Table 6).

### 3.6. Relationship between NGAL, ECP, and Allergy-Related Parameters

After adjusting for potential confounders, NGAL was positively correlated with TNF-*α* (*r* = 0.332), TGF-*β*1 (*r* = 0.285), and hsCRP (*r* = 0.413), but not with ECP, IL-5, and tIgE (Table 7).

Scatter plots of the relationship between NGAL and TGF-*β*1 in patients with bronchial asthma and the relationship between ECP and IL-5 in allergic patients are shown in Figure 2. NGAL and ECP were positively correlated with TGF-*β*1 (*y* = 0.009*x* + 1.436, *r*^2^ = 0.127, *P* < 0.001) and IL-5 (*y* = 0.029*x* + 13.761, *r*^2^ = 0.102, *P* < 0.001), respectively (Figure 2).

### 3.7. Odds Ratio for High TGF-*β*1 with NGAL Elevation

To determine whether NGAL elevation is associated with the prevalence of high TGF-*β*1, multivariate logistic regression analysis was performed. An elevated NGAL level (>150 ng/mL) resulted in a 1.3 times increase in the prevalence of high TGF-*β*1 with adjustment for confounders (odds ratio: 1.31, 95% CI: 1.04–2.58, *P* < 0.001) (Table 8).

## 4. Discussion

In the present study, the relationship between NGAL, ECP, cytokines, sIgE, tIgE, and hsCRP was investigated in patients with allergic diseases. The major findings of this study were as follows: (1) NGAL production was enhanced in allergies; however, increased NGAL production was not associated with a positive ECP test and a high sIgE score; (2) allergic patients without systemic inflammation did not differ from healthy individuals in terms of NGAL; and (3) NGAL was closely associated with TGF-*β*1 and TNF-*α*, but not with ECP and sIgE. These findings are in accordance with the results of a previous study, which demonstrated that NGAL was a prognostic biomarker in asthma-COPD overlap syndrome characterized by airway inflammation [18].

Atopic sensitization refers to a condition with an increased sIgE level after exposure to allergens. It is usually defined as an increase in the concentration to ≥0.35 kU/L of sIgE in response to the corresponding allergens [17]. The sIgE is fundamental to the pathogenesis of allergic disorders, with the relationship between the serum IgE level and the severity of allergic diseases reported widely. In one study, serum IgE levels were significantly higher in asthmatic patients with decreased lung function than in those without decreased lung function [19]. Wood et al. [20] demonstrated that sIgE levels were significantly correlated with both pulmonary function and asthmatic symptoms in patients with inhalant allergies. The present study evaluated whether the plasma NGAL level is more elevated in patients with severe sensitization than in those with mild sensitization. In our study, no significant difference was noted in NGAL concentrations between patients with high and low sIgE scores. These results suggest that the severity of atopic sensitization has no meaningful effect on NGAL elevation in patients with allergic diseases.

ECP can induce epithelial cell death via necrosis and apoptosis pathways [21, 22]. The administration of recombinant ECP triggers smooth muscle cell death within 1 h [23]. The blood ECP level represents the extent of eosinophil activation. Recently, several studies reported that the ECP/Eo ratio is a better indicator for assessing eosinophil activation than ECP [24, 25]. Fujitaka et al. [25] reported that the ECP/Eo ratio was more closely correlated with the clinical symptoms of asthmatic patients than ECP and eosinophil counts. In our study, NGAL production in allergic diseases was evaluated in relation to ECP levels and the ECP/Eo ratio. NGAL levels did not differ between the groups categorized by the ECP level and ECP/Eo ratio. However, the plasma NGAL level was two-fold higher in patients with a positive ECP test and hsCRP elevation than in those with a positive ECP test without hsCRP elevation. These results imply that NGAL may not be elevated in the early phase of allergies, in which ECP is released regionally from activated eosinophils, but systemic inflammation is still not evident. However, NGAL appears to rise as allergies progress, particularly when allergies are accompanied by systemic inflammation. Therefore, it is believed that NGAL elevation in allergies may be suggestive of the advanced or complicated state associated with neutrophilic inflammation.

Activated neutrophils release NGAL and matrix metalloproteinase 9 (MMP-9). NGAL binds to MMP-9 and prevents its inactivation, which leads to the increased degradation of matrix proteins and extended effects on collagen breakdown [26, 27]. Several studies reported that NGAL and MMP-9 levels were increased in the bronchoalveolar lavage samples of patients with asthma as a result of structural alterations in the airways [28, 29]. TGF-*β*1 is a profibrotic cytokine associated with airway fibrosis, playing an essential role in most of the cellular biological processes leading to airway remodeling [30]. In our study, TGF-*β*1 was measured in patients with bronchial asthma to assess any possible relationship between NGAL and the structural alteration of the airway system. Patients with elevated NGAL exhibited higher TGF-*β*1 levels than those without elevated NGAL, and NGAL was positively correlated with TGF-*β*1 even after adjustment for confounders. Multivariate logistic regression analysis also revealed that an elevated NGAL level was closely associated with the prevalence of high TGF-*β*1. These results are in agreement with those of previous studies, showing that TGF-*β*1 expression was upregulated in bronchial asthma [31], and NGAL levels were higher in asthmatic patients with an obstructive ventilatory defect than in those without an obstructive ventilatory defect [32]. These findings indicate that NGAL elevation in patients with asthma may reflect an evolution of allergic inflammation into the airway structural alteration, mediated by fibrotic transformation.

IL-5 is a cytokine that stimulates the production of eosinophils in the bone marrow and is mostly secreted from lymphocytes, tumor cells, and eosinophils [33, 34]. IL-5 elevation can induce eosinophilia in circulating blood or tissues by triggering eosinophil production and preventing eosinophil destruction [35]. In our study, the IL-5 level was significantly higher in patients with a positive ECP test than in those with a negative ECP test, demonstrating a positive correlation with ECP. However, in patients with a positive ECP test, there was no significant difference in the IL-5 level between those with and without elevated hsCRP. Based on these results, it is estimated that although IL-5 may be closely associated with ECP production, its elevated level may not play a crucial role in the development of systemic inflammation in allergic diseases.

This study has several limitations. Arterial blood gas analysis was not performed to evaluate the status of hypoxemia, which might affect plasma NGAL level. Tissue biopsy and pulmonary function tests were not performed to examine the pathologic findings of airway fibrosis and obstructive ventilatory defect in asthmatic patients. Our patient group consisted of heterogeneous populations with small sample sizes, and the levels of NGAL, ECP, and cytokines could not be assessed according to the types of allergies. As our investigation was a cross-sectional study, the evidence for a cause-and-effect relationship between NGAL and ECP was limited. Hence, further investigation is required to verify our findings in a larger randomized prospective trial.

## 5. Conclusions

In conclusion, this study demonstrates that augmented NGAL production may be more closely linked to allergic inflammation in conjunction with proinflammatory cytokines than to the intensity of eosinophil activation and the magnitude of atopic sensitization in allergic diseases. High TGF-*β*1 levels were observed in asthmatic patients with elevated NGAL, suggesting that NGAL elevation may be associated with a potential fibrotic change in the airways in bronchial asthma.

## Figures and Tables

**Figure 1:** Plasma NGAL level in patients with allergic diseases and healthy individuals (∗*P* < 0.001).

**Figure 2:** Scatter plots showing the relationship between NGAL and TGF-*β*1 in patients with bronchial asthma (a) and between ECP and IL-5 in allergic patients (b).

**Table 1:** Clinical presentation of patients with allergic diseases.

*Parameters*	Patients with allergic diseases (*n* = 136)
Age (years)	50.2 ± 12.9
Sex (men/women)	71/65
*Allergy history*	
Duration of allergic diseases (years)	1.4 (0.5–3.5)
Patients with allergic attacks (*n*, %)	75 (55.1)
Frequency of attack/year	1.9 (0–6)
*Allergy type (n, %)*	
Inhalant allergy	105 (77.2)
Food allergy	31 (22.8)
*Clinical parameters (n, %)*	
Current smoking	28 (20.6)
Overweight (BMI ≥ 25.0 kg/m^2^)	43 (31.6)
Hypertension	25 (18.4)

Data are expressed as mean ± SD, median (range), or frequency (percentage). BMI: body mass index.

**Table 2:** Clinical and laboratory characteristics of subjects.

Parameters	Patients (*n* = 136)	Healthy subjects (*n* = 58)	*P* value
*Anthropometric parameters*			
Age (years)	50.2 ± 12.9	51.6 ± 12.5	0.485
Sex (male, %)	71 (52.2)	31 (53.4)	0.876
BMI (kg/m^2^)	22.5 ± 3.8	22.7 ± 4.1	0.743
SBP (mmHg)	123.1 ± 7.2	121.5 ± 6.4	0.145
*Lipocalin*			
NGAL (ng/mL)	137.5 (97.5–174.0)	69.5 (50.7–110.5)	<0.001
Elevated NGAL (*n*, %)	56 (41.2)	0 (0.0)	<0.001
*Allergic parameters*			
ECP (*μ*g/L)	46.9 (31.2–87.6)	11.7 (3.5–16.4)	<0.001
ECP/Eo ratio	0.24 (0.05–6.21)	0.08 (0.03–0.42)	<0.001
Elevated ECP (*n*, %)	110 (80.9)	0 (0.0)	<0.001
tIgE (IU/mL)	351.5 (26.0–872.4)	13.8 (4.5–92.1)	<0.001
sIgE score	3 (2–5)	0 (0–0)	<0.001
*Inflammatory markers*			
hsCRP (mg/dL)	1.24 (0.25–3.79)	0.09 (0.06–0.38)	<0.001
Elevated hsCRP (*n*, %)	91 (66.9)	0 (0.0)	<0.001

Data are expressed as mean ± SD, median (IQR), or frequency (percentage). BMI: body mass index; SBP: systolic blood pressure; NGAL: neutrophil gelatinase-associated lipocalin; ECP: eosinophil cationic protein; ECP/Eo ratio: ECP/eosinophil count ratio; tIgE: total immunoglobulin E; sIgE: specific IgE; and hsCRP: high-sensitivity C-reactive protein.

**Table 3:** NGAL levels in allergic patients with and without systemic inflammation.

Parameters	Allergic patients (*n* = 136)		Healthy subjects (*n* = 58)
	With systemic inflammation (*n* = 91)	Without systemic inflammation (*n* = 45)	
*Clinical parameters*			
Age (years)	50.8 ± 12.2	49.7 ± 13.6	51.6 ± 12.5
Sex (male, %)	47 (53.2)	24 (53.3)	31 (53.4)
*Laboratory parameters*			
NGAL (ng/mL)	152.3 (118.5–214.0) ^a,b^	86.7 (59.5–132.0)	69.5 (50.7–110.5)
ECP (*μ*g/L)	47.6 (36.1–90.2)^b^	41.2 (31.0–86.5)^b^	11.7 (3.5–16.4)
ECP/Eo ratio	0.29 (0.08–6.57)^a,b^	0.20 (0.04–5.02)^b^	0.08 (0.03–0.42)
hsCRP (mg/dL)	2.16 (0.61–4.07)^a,b^	0.23 (0.12–0.43)^b^	0.09 (0.06–0.38)
tIgE (IU/mL)	365.1 (27.5–891.4)^b^	320.7 (23.1–854.6)^b^	13.8 (4.5–92.1)
sIgE score	3 (2–5)^b^	3 (2–5)^b^	0 (0–0)

Data are expressed as mean ± SD, median (IQR), or frequency (percentage). ^a^Significant (*P* < 0.05), compared with allergic patients without systemic inflammation. ^b^Significant (*P* < 0.05), compared with healthy subjects. NGAL: neutrophil gelatinase-associated lipocalin; ECP: eosinophil cationic protein; ECP/Eo ratio: ECP/eosinophil count ratio; hsCRP: high-sensitivity C-reactive protein; tIgE: total immunoglobulin E; and sIgE: specific IgE.

**Table 4:** ECP and inflammatory parameters according to the NGAL level in allergic patients.

Parameters	Allergic patients		*P* value
	Elevated NGAL (*n* = 56)	Nonelevated NGAL (*n* = 80)	
*Clinical parameters*			
Age (years)	51.4 ± 13.1	50.6 ± 12.2	0.715
Sex (male, %)	29 (51.7)	38 (47.5)	0.631
*Allergic parameters*			
ECP (*μ*g/L)	58.2 (29.7–96.4)	37.6 (25.8–83.5)	0.172
ECP/Eo ratio	0.31 (0.10–6.53)	0.23 (0.08–5.13)	0.253
tIgE (IU/mL)	381.5 (31.5–893.6)	310.6 (24.3–681.6)	0.214
sIgE score	4 (2–5)	3 (2–5)	0.307
*Inflammatory parameters*			
TNF-*α* (pg/mL)	71.5 (7.3–290.4)	30.8 (6.5–214.6)	<0.001
IL-5 (pg/mL)	14.9 (8.5–28.6)	11.2 (6.4–22.9)	0.568
TGF-*β*1 (ng/mL)∗	3.52 (1.65–4.58)	1.87 (1.03–3.54)	<0.001
hsCRP (mg/dL)	2.13 (0.42–3.27)	0.45 (0.02–1.62)	<0.001

Data are expressed as mean ± SD or median (IQR). ∗TGF-*β*1 was measured in only patients with bronchial asthma. ECP: eosinophil cationic protein; ECP/Eo ratio: ECP/eosinophil count ratio; tIgE: total immunoglobulin E; sIgE: specific IgE; TNF-*α*: tumor necrosis factor-*α*; IL-5: interleukin-5; TGF-*β*1: transforming growth factor-*β*1; hsCRP: high-sensitivity C-reactive protein; and NGAL: neutrophil gelatinase-associated lipocalin.

**Table 5:** NGAL and proinflammatory cytokines in allergic patients according to the ECP level and ECP/Eo ratio.

Parameters	ECP test		ECP/Eo ratio	
	Positive (*n* = 110)	Negative (*n* = 26)	Elevated (*n* = 68)	Nonelevated (*n* = 68)
*Lipocalin*				
NGAL (ng/mL)	140.5 (71.2–183.0)	128.0 (61.5–164.5)	143.5 (80.2–193.7)	131.0 (60.5–171.8)
*Proinflammatory cytokines*				
IL-5 (pg/mL)	15.8 (10.4–29.5)∗	7.3 (5.1–20.6)	16.4 (9.8–30.7)∗	8.7 (4.9–21.4)
TNF-*α* (pg/mL)	52.7 (8.5–281.2)	46.2 (7.6–252.9)	54.1 (9.3–273.1)	48.5 (6.2–265.3)
TGF-*β*1 (ng/mL)	2.76 (1.59–4.61)	2.43 (1.47–3.84)	2.83 (1.52–4.86)	2.47 (1.45–3.96)
*Allergic parameters*				
tIgE (IU/mL)	423.5 (32.6–904.7)∗	212.3 (19.2–650.8)	482.6 (41.3–981.5)∗	210.7 (18.3–612.4)
sIgE score	4 (2–5)∗	2 (1–3)	4 (2–5)∗	2 (1–3)

Data are expressed as median (IQR). ∗Significant (*P* < 0.001), compared with the corresponding group. NGAL: neutrophil gelatinase-associated lipocalin; IL-5: interleukin-5; TNF-*α*: tumor necrosis factor-*α*; TGF-*β*1: transforming growth factor-*β*1; tIgE: total immunoglobulin E; sIgE: specific IgE; ECP: eosinophil cationic protein; and ECP/Eo ratio: ECP/eosinophil count ratio.

**Table 6:** NGAL, ECP, and proinflammatory cytokines according to sIgE and hsCRP levels.

Parameters	sIgE score		Positive ECP test	
	High (*n* = 86)	Low (*n* = 50)	Elevated hsCRP (*n* = 69)	Nonelevated hsCRP (*n* = 41)
*Lipocalin*				
NGAL (ng/mL)	152.0 (75.3–194.0)	128.0 (62.5–171.5)	181.5 (127.0–236.5)∗	90.2 (60.5–143.0)
*Allergic parameters*				
ECP (*μ*g/L)	62.5 (28.7–95.3)∗	31.4 (25.6–58.1)	50.1 (30.6–82.3)	43.2 (29.3–72.8)
ECP/Eo ratio	0.35 (0.15–9.24)∗	0.14 (0.04–5.61)	0.28 (0.13–7.06)	0.23 (0.07–6.84)
*Proinflammatory cytokines*				
IL-5 (pg/mL)	14.3 (7.2–24.6)	12.7 (6.9–23.5)	14.5 (7.0–25.8)	12.9 (6.5–24.1)
TNF-*α* (pg/mL)	55.2 (7.1–263.8)	42.9 (6.5–243.2)	62.8 (10.4–312.6)∗	30.6 (6.4–231.2)
TGF-*β*1 (ng/mL)	2.87 (1.59–4.83)	2.51 (1.49–3.65)	3.49 (1.92–5.08)∗	1.81 (1.24–3.25)

Data are expressed as median (IQR). ∗Significant (*P* < 0.001), compared with the corresponding group. NGAL: neutrophil gelatinase-associated lipocalin; ECP: eosinophil cationic protein; ECP/Eo ratio: ECP/eosinophil count ratio; IL-5: interleukin-5; TNF-*α*: tumor necrosis factor-*α*; TGF-*β*1: transforming growth factor-*β*1; sIgE: specific immunoglobulin E; and hsCRP: high-sensitivity C-reactive protein.

**Table 7:** Relationship between NGAL, ECP, cytokines, and allergy-related parameters.

Parameters	Multivariate regression analysis∗ (*n* = 136)	
	NGAL	ECP
IL-5	0.121 (0.204)	0.264 (<0.001)
TNF-*α*	0.332 (<0.001)	0.145 (0.124)
TGF-*β*1	0.285 (<0.001)	0.157 (0.116)
ECP	0.114 (0.213)	NA
ECP/Eo ratio	0.136 (0.152)	NA
hsCRP	0.413 (<0.001)	0.136 (0.129)
tIgE	0.092 (0.307)	0.327 (<0.001)
sIgE	0.105 (0.221)	0.289 (<0.001)

Data are expressed as standardized *β* (*P* value). ∗Adjusted for age, sex, BMI, SBP, and current smoking. IL-5: interleukin-5; TNF-*α*: tumor necrosis factor-*α*; TGF-*β*1: transforming growth factor-*β*1; ECP: eosinophil cationic protein; ECP/Eo ratio: ECP/eosinophil count ratio; hsCRP: high-sensitivity C-reactive protein; tIgE: total immunoglobulin E; sIgE: specific IgE; NGAL: neutrophil gelatinase-associated lipocalin; and NA: not applicable.

**Table 8:** Elevated NGAL level as a risk factor for the prevalence of high TGF-*β*1 in allergic patients.

Elevated NGAL (>150 ng/mL)	Prevalence of high TGF-*β*1	
	Odds ratio (95% CI)	*P* value
Unadjusted	3.39 (1.19–8.62)	<0.001
*Adjusted for*		
Age and sex	2.35 (1.17–6.05)	<0.001
Age, sex, and BMI	1.83 (1.15–3.92)	<0.001
Age, sex, BMI, and SBP	1.42 (1.08–2.72)	<0.001
Age, sex, BMI, SBP, and current smoking	1.31 (1.04–2.58)	<0.001

NGAL: neutrophil gelatinase-associated lipocalin; BMI: body mass index; SBP: systolic blood pressure; TGF*-β1*: transforming growth factor-*β*1; and CI: confidence interval.

## Data Availability

The data used to support the findings of this study are available on request from the corresponding author.
